The article "Effect of potassium fertilizer on the growth, physiological parameters, and water status of Brassica juncea cultivars under different irrigation regimes" was retracted in 2023. Reasons: unreliable data; unreliable results or conclusions; concerns about the data; concerns about the peer review.

# Effect of potassium fertilizer on the growth, physiological parameters, and water status of *Brassica juncea* cultivars under different irrigation regimes

**DOI:** 10.1371/journal.pone.0257023

**Published:** 2021-09-23

**Authors:** Preeti Rani, Ishan Saini, Narender Singh, Prashant Kaushik, Leonard Wijaya, Amal Al-Barty, Hadeer Darwish, Ahmed Noureldeen

**Affiliations:** 1 Department of Botany, Kurukshetra University, Kurukshetra, Haryana, India; 2 Instituto de Conservación y Mejora de la Agrodiversidad Valenciana, Universitat Politècnica de València, Valencia, Spain; 3 Department of Biology, Institut Teknologi Sumatera, Jalan Terusan Ryacudu, Way Hui, Jati Agung, South Lampung, Indonesia; 4 Department of Biology, College of Sciences, Taif University, Taif, Saudi Arabia; 5 Department of Biotechnology, College of Sciences, Taif University, Taif, Saudi Arabia; Harran Üniversitesi: Harran Universitesi, TURKEY

## Abstract

Abiotic stress, especially a lack of water, can significantly reduce crop yields. In this study, we evaluated the physiological and biochemical effects of potassium sulfate (K_2_SO_4_) fertilizer and varied irrigation regimes on the economically significant oilseed crop, *Brassica juncea* L, under open field conditions. Two cultivars (RH-725 and RH-749) of *B*. *juncea* were used in a randomized complete block design experiment with three replicates. Irrigation regimes consisted of a control (double irrigation: once at the 50% flowering and another at 50% fruiting stages), early irrigation (at 50% flowering only), late irrigation (at 50% fruiting only) and stress (no irrigation). The K_2_SO_4_ applications were: control (K_0_, no fertilization); K_1_, 10 kg ha^−1^; and K_2_, 20 kg ha^−1^. We measured growth via fresh and dry plant weight, plant height, root length, and leaf area. All the growth parameters were higher in RH-749. The physiological attributes, including the membrane stability index and relative water content, were higher at the 50% flowering stage in RH-749. The amount of antioxidant enzymes (catalase (CAT), guaiacol peroxidase (POX), ascorbate peroxidase (APX), and superoxide dismutase (SOD)) was enhanced when both plants were fertilized during water stress. All of these enzymes had higher activity in RH-749. The total chlorophyll content and photosynthesis rate were considerably higher in RH-749, which leaked fewer electrolytes and maintained a less destructive osmotic potential under limited water conditions. The results indicated that it is water-stress tolerant when given a high concentration of K_2_SO_4_, which alleviated the adverse effects of water stress on growth and physiology.

## Introduction

*Brassica juncea* L. (Indian mustard) is an economically important oilseed crop of the Brassicaceae family (mustard family), planted as a rabi (winter) crop mainly in northern and north-western India [1, 2]. As the country’s population increases, so does the demand for oilseed crops. *B*. *juncea* is also used in phytoremediation of heavy metals like cadmium (Cd) and lead (Pb) [3]. *B*. *juncea* is valuable as a cooking oil [4]: 40% vegetable oil by weight with a caloric value of 541 (per 100 g) and a protein content of 38% [5]. It contains potassium (K), phosphorus (P), sodium (Na), iron (Fe), calcium (Ca), vitamin A, thiamine, niacin, glucosinolates (which regulate stress responses such as the formation of antioxidants), and erucic acid, associated with cardiac injury in cattle. As with any crop, the yield of *B*. *juncea* depends highly on environmental conditions and a primary causes of low productivity is abiotic stress from inadequate irrigation and fertilization [1].

Fertilizers, weedicides, fungicides, and pesticides are essential for increasing yields and continuing production throughout the year under optimal or sub-optimal weather conditions [6]. Water stress, an extended period of low precipitation, affects almost 40% of the 6–7 million hectares of farmland in India. Drought affects crop yields globally on a scale that affects the earth’s carbon sink [7–9], and it will become a more severe problem for future farm production. Because populations continue to grow in water-scarce areas, deficit irrigation may be an efficient means to increase productivity. Water stress seriously impairs many physiological and metabolic processes and may also damage flower or seed development and be responsible for yield gaps [10]. Water stress correlates with high-temperature stress, particularly in arid and semi-arid regions like the state of Haryana in India [11].

Plants have evolved several molecular and physiological mechanisms to respond to environmental stresses, and for certain crop plants applying an additional potassium can enhance these responses [12]. Optimizing irrigation and fertilizer application to improve water retention, stomatal conductance, and light absorption, results in increased crop development and yield [13]. Potassium is an essential macronutrient and the most crucial osmoticum for vegetables [14]. It is required for a plant’s mechanical stability, nutrition, development, reproduction, and resistance to pathogens [15]. Applying potassium can help to alleviate abiotic stress by increasing photosynthate translocation and enhancing gas exchange, protein synthesis, enzyme activity, and stomatal conductance [16, 17].

Moreover, potassium reduces water damage and stimulates anti-stress enzyme systems while enlarging the root system. This increases translocation, improves water absorption, reduces respiration, and increases photosynthetic activity, which enhances crop development and decreases lodging [18]. Therefore, we studied the effect of potassium fertilizer on the growth, physiological parameters, and water status of *B*. *juncea* cultivars under different water conditions.

## Materials and methods

### Experimental layout

The field experiment was carried out from October to March 2018–2019 and 2019–2020 at a nursery in Kurukshetra University, Kurukshetra, India (29°95’N; 76°82’E). Day, and night-time temperatures averaged 30 ± 4°C and 20 ± 5°C, respectively. The sandy-clayey loamy soil, was ploughed to create a uniform plot. The experiment was designed as a randomized complete block with a factorial treatment structure in three replicates. The four irrigation regimes induced water stress by withholding irrigation during a vital development stage (siliquae (fruit) development and flower initiation). It consisted of: control (irrigated twice, at the 50% flowering and 50% siliquae formation stages), late stress (once at 50% flowering), early stress (once at 50% siliquae formation), and total stress (no irrigation).

Two *Brassica* cultivars (RH-725 and RH-749) were fertilized at three K_2_SO_4_ levels: K_0_ (0 kg/ha), K_1_ (10 kg/ha), and K_2_ (20 kg/ha), which were applied with the recommended rates of nitrogen (N), phosphorous (P) and K: urea, superphosphate, and potassium sulphate (K_2_SO_4_), respectively (Table 1). The seeds were obtained from the oilseed section of Chaudhary Charan Singh Hisar Agricultural University, Haryana. Previous physicochemical analysis of the soil showed that it consisted of 80.32% sand, 6.11% silt, 13.18% clay, 0.79% organic matter. The chemical content (kg/ha) were N, 110.15; P 7.59; K 439.61; and 106.49 sulphur (S) [19]. The soil pH was slightly basic at 7.9.

**Table 1:** The 12 treatments in the experiment.

Treatment no.	Treatment code	Treatment details
**T**_**1**_	C + K_0_*	Control (2 irrigations: first at 50% flowering stage; second at 50% siliquae formation time) + K_0_
**T**_**2**_	C + K_1_*	Control (2 irrigations: first at 50% flowering stage; second at 50% siliquae formation time) + K_1_
**T**_**3**_	C + K_2_*	Control (2 irrigations: first at 50% flowering stage; second at 50% siliquae formation time) + K_2_
**T**_**4**_	EI + K_0_	Early irrigation (irrigation at 50% flowering stage only) + K_0_
**T**_**5**_	EI + K_1_	Early irrigation (irrigation at 50% flowering stage only) + K_1_
**T**_**6**_	EI + K_2_	Early irrigation (irrigation at 50% flowering stage only) + K_2_
**T**_**7**_	LI + K_0_	Late irrigation (irrigation at 50% fruiting stage only) + K_0_
**T**_**8**_	LI + K_1_	Late irrigation (irrigation at 50% fruiting stage only) + K_1_
**T**_**9**_	LI + K_2_	Late irrigation (irrigation at 50% fruiting stage only) + K_2_
**T**_**10**_	S + K_0_	Stress (no irrigation) + K_0_
**T**_**11**_	S + K_1_	Stress (no irrigation) + K_1_
**T**_**12**_	S + K_2_	Stress (no irrigation) + K_2_

* K = kg ha^–1^ K_2_SO_4_: K_0_ = 0; K_1_ = 10; K_2_ = 20.

### Plant characterization and data analysis

At the flowering stage (day 65), we measured the root and shoot lengths and calculated the whole plant height. The roots were then separated from the shoot, blow-dried, and weighed to record their fresh weight (FW). They were then placed in an oven at 80°C overnight and weighed again to record their dry weight (DW). According to the manufacturer’s instructions, the leaf area was measured using a portable leaf area meter (Systronics 211, Ahmedabad, India). Plants were harvested at maturity, and plant samples were collected from each plot at the flowering stage. The fresh and dry weights of leaves were measured as described above, and the water content was calculated according to the following equation: Leaf water content = ((FW−DW)/FW) × 100.

### Physiological and biochemical attributes

Chlorophyll content was measured using a CL-01 Chlorophyll Content Meter (Hansateh, Norfolk, UK) that absorbed two wavelengths of light (620 and 940 nm). The membrane stability index (MSI) was measured using methods described by Ali et al. [20]. Two similarly sized leaf disks (200 mg) were briefly collected and placed in test tubes containing 20 mL of double-distilled water. One test-tube was kept at 40°C for 30 min then cooled to 25°C before measuring the initial conductivity (C1) using a conductivity meter. Another test tube was placed in a boiling water bath (100°C) for 15 min and then cooled to 25°C before measuring conductivity (C2). The osmotic potential was measured on the third completely expanded leaf placed in tightly stoppered glass tubes and heated at 45°C for 1 hour to soften the tissue and remove turgidity. The tissue was crushed with a glass rod and placed on a filter paper disc on a concave depression holder. The osmometer was calibrated using the reference standards of sodium chloride and used to measure each sample’s osmotic potential.

Electrolyte leakage was measured as described by Dionisio-Sese and Tobita [21]. Briefly, a fresh leaf was immersed in a test tube containing deionized water. One tube was unheated, another was heated at 50–60°C for about 25 min, and the last at 100°C for 10 min. The electrical conductivities from leachates produced in the unheated (ECa) and heated (ECb), and (ECc) tubes were measured using an electrical conductivity meter.

### Stress parameters and enzymatic assay

To understand how the plants respond to stress, we evaluated the antioxidant defence system comprising peroxidase (POD), ascorbate peroxidase (APX), superoxide dismutase (SOD), and catalase (CAT). Briefly, 0.5 g of fresh leaves was homogenized with 100 mM Tris-HCl, 5.0 mM dithiothreitol, 10 mM magnesium chloride 5.0 mM magnesium acetate, 1.5% polyvinyl pyrrolidone (PVP)-40 and 1.0 mM EDTA. POX was extracted with a 0.01 M phosphate buffer. SOD activity was measured based on the conversion of nitroblue tetrazolium to formazan [22]. CAT activity was measured after the addition of 3 mL of 20 mM H_2_O_2_ in 50 mM phosphate buffer [23]. APX activity was measured based on the decrease in absorbance at 290 nm due to ascorbic acid oxidation [24] (One enzyme unit was defined as the amount of enzyme required to oxidize 1 mole of ascorbic acid per min.) Glutathione reductase was measured using Halliwell and Foyer [25], which involved measuring the oxidation of NADPH by Glutathione reductase at 340 nm. The rate (μmoles min^−1^) was calculated using the extinction coefficient of 6.12 mM^−1^ cm^−1^.

### Statistical analysis

Randomized complete block design (RCBD) was employed with three replications for two different cultivars of *B*. *juncea* (RH-725 and RH-749) under four irrigation schedules. Furthermore, the plants were supplied with varied amounts of K_2_SO_4_. Therefore, the data were analysed for three factors using the OPSTAT software (CCSHAU, Hisar). The critical difference (CD) was calculated at a 5% level of significance for comparing the means.

## Results

The higher application rate of K_2_SO_4_ significantly improved the morphological traits of both *B*. *juncea* cultivars under low water conditions, including water stress. For example, the plant FW, DW, leaf area, and height were all higher in treatments with the highest concentration of K_2_SO_4._ (Table 2). They were also significantly compared to the treatments without K_2_SO_4_, irrespective of irrigation level. Furthermore, the dry matter content of plants grown under late and no irrigation were also similar. The plants with the lowest dry matter contents were the following treatments: S + K_0_, LI + K_0_, and C + K_0_. The dry matter content of both cultivars were comparable except under stress conditions, where cultivar RH-749 performed better. The longest roots (21.7 cm) were measured in C + K_2_ and EI + K_2_, whereas the shortest were found in treatment S + K_0_. Overall, RH-749 had longer roots than RH-725. Measurements of leaf area and plant height were the highest in treatments C + K_2_ and EI + K_2_, while the lowest measurements were found in treatment S + K_0_ (Fig 1). No irrigation generated the highest osmotic potential in treatments S + K_0_, S + K_1_, and S + K_2_, whereas the treatments with higher dosages of K_2_SO_4_ (C + K_2_, EI + K_2_, and LI + K_2_) generated the lowest osmotic potentials.

**Fig 1:** Mean values of fresh weight (colour, g), leaf area (cm^2^) and plant height (cm) of the 12 treatments with different levels of irrigation (C = Control, EI = Early irrigation, LI = Late irrigation, S = Stress) and different amounts of K (kg ha^–1^ K_2_SO_4_): K_0_ = 0; K_1_ = 10; K_2_ = 20.

**Table 2:** Effects of irrigation regime and potassium fertilizer on morphological traits of *Brassica juncea* cultivars.

Treatments*	Dry matter (g)			Root length (cm)			Osmotic potential (MPa)		
	RH-725	RH-749	Mean	RH-725	RH-749	Mean	RH-725	RH-749	Mean
C + K_0_	4.25 ± 0.486^d^	4.39 ± 0.636^d^	4.32 ± 0.375^e^	16.03 ± 0.597^d^	17.38 ± 1.735^f^	16.72 ± 1.526^e^	0.684± 0.412^de^^‡^	0.578 ± 0.865^f^	0.631 ± 0.045^d^
C + K_1_	5.27 ± 0.379^c^	6.02 ± 0.824^c^	5.65 ± 0.528^d^	16.3 ± 0.835^d^	18.44 ± 1.397^e^	17.24 ± 1.497^d^	0.574 ± 0.633^f^	0.521 ± 0.453^f^	0.548 ± 0.454^e^
C + K_2_	12.1 ± 0.176^ab^	12.86 ± 1.188^ab^	12.49 ± 0.833^b^	20.72 ± 0.473^a^	22.76 ± 1.282^a^	21.74 ± 1.914^a^	0.523 ± 0.595^f^	0.479 ± 0.682^g^	0.501 ± 0.127^e^
EI + K_0_	4.55 ± 0.385^d^	5.2 ± 1.034^d^	4.88 ± 0.736^e^	15.35 ± 1.976^e^	16.36 ± 0.649^g^	15.82 ± 1.277^f^	0.738 ± 0.377^d^	0.675 ± 0.576^de^	0.707 ± 0.424^c^
EI + K_1_	5.65 ± 1.034^c^	6.25 ± 0.524^c^	5.95 ± 0.517^d^	18.37 ± 1.622^b^	20.36 ± 0.533^c^	19.32 ± 0.423^b^	0.643 ± 0.583^e^	0.634 ± 0.398^e^	0.639 ± 0.598^d^
EI + K_2_	13.49 ± 0.975^a^	13.81 ± 0.371^a^	13.65 ± 0.423^a^	21.22 ± 1.738^a^	22.36 ± 0.688^a^	21.74 ± 0.287^a^	0.623 ± 0.476^e^	0.628 ± 0.484^e^	0.626 ± 0.374^d^
LI + K_0_	3.09 ± 0.487^e^	3.15 ± 0.536^e^	3.12 ± 0.253^f^	15.32 ± 0.538^e^	15.71 ± 0.534^h^	15.56 ± 0.196^f^	0.835 ± 0.393^cd^	0.758 ± 0.188^c^	0.797 ± 0.936^bc^
LI + K_1_	4.57 ± 0.428^d^	4.82 ± 1.045^d^	4.69 ± 0.414^e^	17.36 ± 0.494^c^	18.34 ± 0.696^e^	17.74 ± 1.064^d^	0.756 ± 0.876^d^	0.727 ± 0.494^c^	0.742 ± 0.094^c^
LI + K_2_	10.34 ± 0.385^b^	11.26 ± 1.634^ab^	10.82 ± 1.832^c^	21.22 ± 0.727^a^	21.42 ± 0.488^b^	21.33 ± 0.758^a^	0.689 ± 0.273^e^	0.675 ± 0.939^de^	0.682 ± 0.518^cd^
S + K_0_	3.06 ± 0.399^e^	2.92 ± 1.073^f^	2.99 ± 1.635^g^	13.37 ± 1.594^f^	15.79 ± 0.414^h^	14.51 ± 0.427^g^	1.045 ± 0.735^a^	0.985 ± 1.045^a^	1.015 ± 0.295^a^
S + K_1_	4.12 ± 0.287^d^	4.93 ± 0.436^d^	4.52 ± 1.836^e^	15.35 ± 1.356^e^	18.55 ± 1.837^e^	16.73 ± 0.593^e^	0.937 ± 0.837^b^	0.904 ± 1.674^a^	0.921 ± 0.427^ab^
S + K_2_	10.18 ± 0.293^b^	11.22 ± 0.520^ab^	10.72 ± 0.638^c^	18.51 ± 1.933^b^	19.31 ± 1.294^d^	18.73 ± 0.388^c^	0.859 ± 0.347^cd^	0.845 ± 0.263^b^	0.852 ± 0.044^b^

*C = Control, EI = Early irrigation, LI = Late irrigation, S = Stress,

^‡^values in columns followed by the same letter are not significantly different, *p* ≤ 0.05, LSD.

The FWs of the control irrigation treatment with the high dosage of K_2_SO_4_ (87 g) and that of the early irrigation treatment with the high dosage of K_2_SO_4_ (88 g) were very similar. The plants with the lowest FWs were those treated with the lower dosages of K_2_SO_4_ in EI + K_0_ (18 g), LI + K_0_ (16 g), and S + K_0_ (14 g) (Fig 1).

The maximum relative water content was observed in cultivar RH-749, in treatment C + K_2_ (85.05%); in this cultivar, the lowest relative water content was observed for treatment S + K_0_ (69.74%) (Fig 2).

**Fig 2:** Mean values of the relative water content (%), membrane stability index (%) and electrolytic content (%) of the 12 treatments with different levels of irrigation (C = Control, EI = Early irrigation, LI = Late irrigation, S = Stress) and different amounts of K (kg ha^–1^ K_2_SO_4_): (K_0_ = 0; K_1_ = 10; K_2_ = 20).

In general, cultivar RH-749 performed better in the vegetative growth parameters. Membrane stability index values of 73.16 and 71.27% were recorded in the treatments C + K_2_ and EI + K_2_, respectively, while the lowest values (56.54 and 59.14%) were found in treatments S + K_0_ and S + K_1_, respectively (Fig 2). The highest level of electrolyte leakage occurred in treatments without irrigation, i.e., S + K_0_, S + K_1_, and S + K_2_, whereas the lowest levels of electrolyte leakage occurred with higher amounts of K_2_SO_4_ (C + K_2_, EI + K_2_, and LI + K_2_) (Fig 2).

The results in Table 3 revealed that the levels of all the antioxidant enzymes increased in the leaves of both *B*. *juncea* cultivars under stress conditions, but were significantly higher in the more water-stress-tolerant RH 749. Specifically, the highest activities of SOD (U g^-1^ FW) were recorded in treatments S + K_2_ (26.59 U g^-1^ FW), LI + K_2_ (23.68 U g^-1^ FW), and EI + K_2_ (22.01 U g^-1^ FW), whereas the lowest was measured in treatment C + K_0_ (14.89 Ug^-1^ FW). APX activities were highest under stress conditions in treatments S + K_2_ (10.31 U g^-1^ FW), S + K_1_ (9.67 U g^-1^ FW), and S + K_0_ (8.80 U g^-1^ FW) (Table 3). Surprisingly, the ascorbate peroxidase activities of treatments LI + K_1_ (4.02 U g^-1^ FW) and LI + K_2_ (4.71 U g^-1^ FW) were less than 50% that of the highest ascorbate peroxidase activities (Table 4). The findings for catalase activity (Table 3) were similar to those of ascorbate peroxidase. The highest catalase activities were observed under stress conditions in treatments S + K_2_ (15.35 U g^-1^ FW), S + K_1_ (11.86 U g^-1^ FW), and S + K_0_ (7.88 U g^-1^ FW). In contrast, the lowest activities were observed for treatments LI + K_1_ (3.60 U g^-1^ FW) and LI + K_2_ (4.22 U g^-1^ FW) (Table 3).

**Table 3:** Effects of irrigation regime and potassium fertilizer on antioxidant activity of *Brassica juncea* cultivars.

Treatments*	Superoxidase dismutase (U g^−1^ FW)			Peroxidase (U g^−1^ FW)			Ascorbate Peroxidase (U g^−1^ FW)			Catalase (U g^−1^ FW)		
	RH-725	RH-749	Mean	RH-725	RH-749	Mean	RH-725	RH-749	Mean	RH-725	RH-749	Mean
C + K_0_	12.62 ± 0.545^i^^‡^	17.16 ± 0.785^h^	14.89 ± 0.756^h^	4.16 ± 1.455^h^	8.17 ± 0.375^h^	15.60 ± 0.544^i^	2.75 ± 0.055^h^	6.83 ± 0.496^h^	5.85 ± 0.485^f^	2.03 ± 0.676^j^	4.36 ± 0.546^j^	5.24 ± 1.198^e^
C + K_1_	13.25 ± 0.387^h^	18.52 ± 0.376^g^	15.89 ± 0.645^g^	5.02 ± 1.856^g^	10.25 ± 0.457^g^	16.71 ± 1.275^g^	4.31 ± 0.156^g^	7.31 ± 0.276^gh^	6.27 ± 0.377^e^	3.12 ± 0.457^i^	4.98 ± 0.857^i^	5.61 ± 1.036^e^
C + K_2_	14.83 ± 0.598^h^	21.68 ± 0.488^f^	18.26 ± 0.427^f^	5.56 ± 1.158^g^	11.52 ± 1.634^f^	19.33 ± 0.856^f^	4.98 ± 0.534^g^	9.59 ± 0.329^g^	7.25 ± 0.948^d^	3.76 ± 0.544^h^	6.73 ± 0.745^h^	6.49 ± 0.578^d^
EI + K_0_	11.75 ± 1.074^i^	18.48 ± 0.535^g^	15.12 ± 0.535^g^	9.63 ± 1.474^de^	13.75 ± 1.887^e^	16.17 ± 0.587^h^	6.55 ± 0.945^f^	8.62 ± 0.457^f^	6.06 ± 0.635^e^	4.25 ± 0.647^gh^	6.59 ± 0.548^h^	5.43 ± 0.860^e^
EI + K_1_	16.21 ± 0.646^e^	22.34 ± 0.587^e^	19.28 ± 1.748^d^	13.21 ± 1.677^c^	15.45 ± 0.647^d^	20.23 ± 0.494^e^	9.62 ± 0.647^d^	11.08 ± 0.785^e^	7.59 ± 0.427^d^	5.51 ± 1.853^gh^	8.92 ± 0.638^gh^	6.80 ± 0.387^d^
EI + K_2_	18.33 ± 0.578^d^	25.68 ± 0.374^de^	22.01 ± 1.937^bc^	14.65 ± 1.577^c^	17.58 ± 0.294^c^	23.15 ± 1.748^c^	10.29 ± 0.585^cd^	13.77 ± 0.218^d^	8.68 ± 0.582^c^	7.82 ± 0.567^fg^	10.18 ± 0.655^g^	7.78 ± 0.644^c^
LI + K_0_	13.65 ± 0.385^g^	23.11 ± 0.858^e^	18.38 ± 1.673^e^	7.36 ± 0.368^f^	12.55 ± 1.057^f^	19.86 ± 1.949^f^	7.52 ± 0.694^e^	9.72 ± 0.576^e^	7.45 ± 0.545^d^	8.21 ± 0.954^f^	9.02 ± 0.567^f^	6.67 ± 0.396^d^
LI + K_1_	15.58 ± 0.844^f^	25.18 ± 0.812^de^	20.38 ± 1.575^bc^	8.16 ± 0.474^de^	13.26 ± 1.685^e^	10.71 ± 1.844^j^	11.67 ± 0.587^cd^	13.61 ± 0.938^d^	4.02 ± 0.648^g^	10.26 ± 1.057^d^	11.53 ± 0.388^d^	3.60 ± 0.947^g^
LI + K_2_	19.82 ± 0.478^c^	27.53 ± 0.475^c^	23.68 ± 1.436^bc^	10.75 ± 0.833^d^	14.38 ± 0.474^e^	12.57 ± 1.596^h^	14.73 ± 0.855^c^	16.58 ± 0.485^c^	4.71 ± 0.937^g^	12.57 ± 1.268^b^	15.17 ± 0.576^b^	4.22 ± 0.598^f^
S + K_0_	18.16 ± 0.245^d^	26.24 ± 0.339^d^	22.20 ± 1.365^c^	11.98 ± 0.475^d^	15.88 ± 0.288^d^	23.46 ± 0.497^d^	9.52 ± 0.687^d^	11.17 ± 0.858^e^	8.80 ± 0.635^c^	9.52 ± 1.098^e^	10.05 ± 0.247^e^	7.88 ± 0.588^c^
S + K_1_	21.19 ± 0.574^ab^	28.19 ± 1.475^b^	24.69 ± 1.439^b^	19.58 ± 1.736^b^	20.82 ± 0.684^b^	25.78 ± 0.655^b^	15.12 ± 0.454^b^	18.19 ± 0.645^b^	9.67 ± 0.597^b^	11.16 ± 0.675^c^	12.56 ± 0.588^c^	11.86 ± 0.274^b^
S + K_2_	23.68 ± 0.939^a^	29.49 ± 1.938^a^	26.59 ± 1.934^a^	21.62 ± 0.424^a^	22.52 ± 0.483^a^	27.49 ± 0.487^a^	17.08 ± 0.937^a^	20.11 ± 0.578^a^	10.31 ± 0.654^a^	13.17 ± 0.957^a^	17.52 ± 0.387^a^	15.35 ± 0.487^a^

*C = Control, EI = Early irrigation, LI = Late irrigation, S = Stress,

^‡^values in columns followed by the same letter are not significantly different, *p* ≤ 0.05, LSD.

**Table 4:** Effects of irrigation regime and potassium fertilizer on chlorophyll and carotenoid contents of *Brassica juncea* cultivars.

Treatments*	Chlorophyll a (mg g^-1^ FW)			Chlorophyll b (mg g^-1^ FW)			Total chlorophyll (mg g^-1^ FW)			Carotenoid (mg g^-1^ FW)		
	RH-725	RH-749	Mean	RH-725	RH-749	Mean	RH-725	RH-749	Mean	RH-725	RH-749	Mean
C + K_0_	2.76 ± 0.754^ab^^‡^	3.03 ± 0.676^b^	2.90 ± 0.597^b^	0.94 ± 0.245^b^	1.12 ± 0.463^b^	1.03 ± 0.435^b^	3.71 ± 0.476^b^	4.16 ± 0.264^b^	3.93 ± 0.344^b^	0.23 ± 0.656^h^	0.39 ± 0.254^h^	0.31 ± 0.593^h^
C + K_1_	2.83 ± 0.635^ab^	3.21 ± 0.698^b^	3.02 ± 0.534^ab^	0.95 ± 0.734^b^	1.15 ± 0.266^b^	1.05 ± 0.377^b^	3.78 ± 0.746^ab^	4.37 ± 0.674^ab^	4.08 ± 0.653^a^	0.45 ± 0.753^f^	0.51 ± 0.586^ef^	0.48 ± 0.686^f^
C + K_2_	2.97 ± 0.954^a^	3.36 ± 1.085^a^	3.17 ± 0.237^a^	1.01 ± 0.343^a^	1.21 ± 0.438^a^	1.11 ± 0.466^a^	3.98 ± 0.548^a^	4.57 ± 0.384^a^	4.28 ± 0.237^a^	0.87 ± 0.837^b^	0.89 ± 0.487^b^	0.88 ± 0.268^b^
EI + K_0_	2.58 ± 0.648^cd^	2.69 ± 0.697^c^	2.64 ± 0.944^c^	0.86 ± 0.125^bc^	0.87 ± 0.166^bc^	0.86 ± 0.275^c^	3.44 ± 0.578^c^	3.56 ± 0.187^c^	3.50 ± 0.566^c^	0.38 ± 0.935^g^	0.39 ± 0.277^g^	0.39 ± 0.385^g^
EI + K_1_	2.61 ± 0.698^cd^	2.72 ± 0.124^c^	2.67 ± 0.247^d^	0.87 ± 0.464^d^	0.88 ± 0.344^d^	0.88 ± 0.437^d^	3.49 ± 0.765^d^	3.61 ± 0.475^d^	3.55 ± 0.544^d^	0.48 ± 0.856^f^	0.50 ± 0.684^ef^	0.49 ± 0.594^f^
EI + K_2_	2.66 ± 0.454^cd^	2.75 ± 0.286^c^	2.71 ± 0.38^cd^	0.89 ± 1.056^d^	0.92 ± 0.386^cd^	0.90 ± 0.645^cd^	3.56 ± 0.374^cd^	3.67 ± 0.453^cd^	3.61 ± 0.475^cd^	0.90 ± 0.585^b^	0.92 ± 0.663^b^	0.91 ± 0.577^b^
LI + K_0_	2.21 ± 0.576^ef^	2.24 ± 0.476^f^	2.25 ± 0.476^f^	0.72 ± 1.856^f^	0.81 ± 0.547^f^	0.76 ± 0.479^f^	2.94 ± 0.596^f^	3.10 ± 0.685^f^	3.02 ± 0.876^f^	0.42 ± 0.575^f^	0.43 ± 0.386^f^	0.42 ± 0.597^f^
LI + K_1_	2.25 ± 0.785^ef^	2.31 ± 0.588^e^	2.28 ± 0.935^ef^	0.76 ± 0.578^ef^	0.83 ± 0.573^f^	0.80 ± 0.526^f^	3.01 ± 0.587^ef^	3.15 ± 0.238^ef^	3.08 ± 0.597^ef^	0.52 ± 0.376^e^	0.56 ± 0.543^e^	0.54 ± 0.645^e^
LI + K_2_	2.28 ± 0.364^ef^	2.36 ± 0.485^ef^	2.32 ± 0.484^ef^	0.78 ± 0.386^ef^	0.84 ± 0.526^f^	0.81 ± 0.637^f^	3.07 ± 0.587^ef^	3.20 ± 1.736^ef^	3.13 ± 0.476^de^	1.01 ± 0.737^a^	1.56 ± 0.476^a^	1.29 ± 0.586^a^
S + K_0_	2.05 ± 0.346^g^	2.11 ± 0.699^g^	2.08 ± 0.296^g^	0.62 ± 0.375^g^	0.67 ± 0.848^g^	0.65 ± 0.685^g^	2.67 ± 0.645^g^	2.79 ± 1.936^g^	2.73 ± 0.847^g^	0.62 ± 0.584^d^	0.64 ± 0.528^d^	0.63 ± 0.638^d^
S + K_1_	2.26 ± 0.768^ef^	2.32 ± 0.276^e^	2.30 ± 0.776^e^	0.76 ± 0.547^e^	0.82 ± 0.325^e^	0.79 ± 0.797^e^	3.02 ± 0.958^e^	3.14 ± 0.526^e^	3.08 ± 0.587^e^	0.76 ± 0.486^c^	0.81 ± 0.578^c^	0.78 ± 0.386^c^
S + K_2_	2.31 ± 0.266^e^	2.45 ± 0.598^d^	2.38 ± 0.584^d^	0.77 ± 0.384^cd^	0.83 ± 0.527^d^	0.80 ± 0.535^d^	3.09 ± 0.864^de^	3.28 ± 0.636^d^	3.18 ± 0.668^d^	1.34 ± 0.577^a^	1.78 ± 0.635^a^	1.56 ± 0.648^a^

*C = Control, EI = Early irrigation, LI = Late irrigation, S = Stress,

^‡^values in columns followed by the same letter are not significantly different, *p* ≤ 0.05, LSD.

In Table 4, decreasing water availability resulted in decreased chlorophyll a and b. However, carotenoid levels increased. The highest levels of chlorophyll a were observed in treatments C + K_2_ (3.17 mg g^-1^ FW), C + K1 (3.02 mg g^-1^ FW), and EI + K_2_ (2.71 mg g^-1^ FW), with the highest chlorophyll b levels occurring in the same treatments at concentrations of 1.11, 1.05, and 0.90 mg g^-1^ FW, respectively. Meanwhile, the lowest levels of total chlorophyll (chlorophylls a + b) were observed in treatments S + K_0_ (2.73 mg g^-1^ FW), LI + K_0_ (3.02 mg g^-1^ FW), and LI + K_1_ (3.08 mg g^-1^ FW). The highest carotenoid levels were observed in treatments S + K_2_ (1.56 mg g^-1^ FW), LI + K_2_ (1.29 mg g^-1^ FW), and EI + K_2_ (0.91 mg g^-1^ FW), while the lowest levels were observed in treatments C + K_0_ (0.31 mg g^-1^ FW), EI + K_0_ (0.39 mg g^-1^ FW), and LI + K_0_ (0.42 mg g^-1^ FW) (Table 4). Overall, cultivar RH-749 showed higher contents of chlorophyll and carotenoids than RH-725.

## Discussion

Among the abiotic stresses, the lack water has the most severe effects on crop growth and yield, and plants must adapt to water stress to survive. The bulk of the potassium requirement of plants, used to maintain average growth and development, is absorbed from the soil [26, 27]. Excess or deficiency in potassium hampers the plant’s overall growth [28] because it is required for various biochemical and physiological processes, including protein synthesis, carbohydrate metabolism, and enzyme activation [29].

During water stress, a plant’s water potential is decreased to the extent that cellular activity is hampered [30]. By disturbing the water potential, any abiotic stress can reduce crop cellular activities during the flowering and grain filling stages. Fertilizers, particularly potassium, play a significant role in adjusting the osmotic potential [14]. It also plays a role in many fundamental processes, such as nitrogen use, protein biosynthesis, cell growth, cell expansion (by stimulating gibberellins), and overall plant development. Thus, plant FW, DW, leaf area, and plant height were significantly higher in RH-749 [31, 32]. Potassium plays a role in increasing the efficiency of chlorophyll (the main component of chloroplasts), thereby increasing photosynthesis. The formation of carbohydrates was accelerated in our experimental treatments where potassium fertilizer was added [33, 34]. Potassium also increases carotenoid levels during stress, possibly by inhibiting the proteins (porins and transporter) in the thylakoid membranes of the chloroplast [34, 35]. This may be why total chlorophyll and carotenoid levels in treatments increased more in RH-749 than RH-725. These previous works indicated that potassium can accelerate enzymatic biochemical reactions and encourage early growth, which supports our findings [30, 32, 35]. For example, potassium influences the transport of sap and expansin proteins [36, 37]. In another example, it was reported to have helped loosen cell walls by activating the ATPase pump that generates acidic conditions in the periplasmic space [38].

As mentioned above, potassium can modify the utilization of nitrogen, the most abundant element in the earth’s atmosphere and plays a significant role in crop maturation, especially during fruit development [39, 40]. Nitrate acquisition is frequently correlated with potassium fertilizer (K_2_SO_4_), resulting in enhanced amino acids and proteins [31]. As a mobile element, potassium also regulates osmotic pressure and maintains ionic stability within the cytoplasm [41]. The various roles potassium plays are related to the opening and closing of stomata and other physiological processes [41]. This explains why, in plants treated with potassium, the osmotic potential, relative water content, membrane stability index, and electrolytic content increased [42, 43]. Others have reported that potassium induces the enhancement of proline, a substance that responds to stress and regulates osmotic and turgor pressure [44, 45]. Potassium helps maintain the electrical balance within cells, specifically at the site of ATP synthesis and is responsible for controlling the opening and closing of guard cells, thus regulating photosynthesis [46, 47]. The involvement of potassium in all these processes explains why electrolyte leakage and osmotic potential were lower in RH-749 treatments than those for RH-725. Water conductivity and photosynthetic efficiency were also higher. Potassium fertilizers are also known to help fruit development in *Malus domestica* and *Pyrus* [48, 49].

The higher application rates of K_2_SO_4_ significantly improved the morphological traits of both *B*. *juncea* cultivars under low water conditions, including water stress. Similarly, Hu, Jiang [50] reported increased levels of stress response-related enzymes. Potassium is a cofactor in various enzymatic reactions in carbohydrate biosynthesis, photosynthesis, and stress regulation [51]. CAT (a tetrameric haem-containing enzyme) detoxifies reactive oxygen species by converting hydrogen peroxide into water [52], while POD mainly oxidizes OH free radicals into H_2_O [53]. Ascorbic acid-dependent APX is the only enzyme capable of scavenging H_2_O_2_ in the chloroplast, where CAT is not present [35]. Akram, Iqbal [54] confirmed that CAT and POD were upregulated in two cultivars of *B*. *napus* upon exposure to water deficit conditions. Research by Al Mahmud, Hasanuzzaman [55] showed that *B*. *juncea* forms ascorbic acid and CAT in response to cadmium toxicity while synthesizing dehydroascorbate reductase (DHAR), SOD, monodehydroascorbate reductase (MDHAR), and GR upon potassium application. The application of potassium also mitigates water stress in many other crop plants such as *Nicotiana rustica*, *Zea mays*, and *Oryza sativa* [32, 45, 56]. Potassium also alleviates salt stress because it is, directly and indirectly, involved in antioxidant activation, an adaptive salt-stress response [57]. Furthermore, potassium also regulates plant development by augmenting the flavonoids, phenolics, polyphenols, antioxidants, and secondary metabolites of plants during stress [58].

## Conclusion

Our results show varietal differences in *B*. *juncea* responses to potassium application. When treated with optimal potassium levels, RH-749 had i) higher water-holding efficiency, ii) enhanced photosynthesis, iii) upregulated enzymatic activity, iv) less electrolytic leakage, and v) improved overall development compared to RH-725. Although potassium is an essential nutrient, it is not involved in the physiological functions mentioned in the paper. However, it improves nitrogen and carbon use efficiency. Potassium and nitrogen, separately or together, affected the yield and quality of *Brassica juncea*. In both cultivars, a high application rate of potassium fertilizer resulted in increased activity of all antioxidant enzymes; however, the maximum responses to potassium under all irrigation regimes were observed in RH-749.

Furthermore, the levels of all the photosynthetic pigments decreased as water stress increased. The maximum pigment levels occurred in the control for all concentrations of potassium. However, these levels were significantly reduced under stress conditions. High application rates for potassium alleviated the negative effect of water stress, as shown by the increased levels of photosynthetic pigments.
